The article "Phenopacket-tools: Building and validating GA4GH Phenopackets" was published in 2023. Journal: PLoS One.

# Phenopacket-tools: Building and validating GA4GH Phenopackets

**DOI:** 10.1371/journal.pone.0285433

**Published:** 2023-05-17

**Authors:** Daniel Danis, Julius O. B. Jacobsen, Alex H. Wagner, Tudor Groza, Martha A. Beckwith, Lauren Rekerle, Leigh C. Carmody, Justin Reese, Harshad Hegde, Markus S. Ladewig, Berthold Seitz, Monica Munoz-Torres, Nomi L. Harris, Jordi Rambla, Michael Baudis, Christopher J. Mungall, Melissa A. Haendel, Peter N. Robinson

**Affiliations:** 1 The Jackson Laboratory for Genomic Medicine, Farmington, CT, United States of America; 2 William Harvey Research Institute, Queen Mary University of London, London, United Kingdom; 3 Departments of Pediatrics and Biomedical Informatics, The Ohio State University College of Medicine, Columbus, OH, United States of America; 4 The Steve and Cindy Rasmussen Institute for Genomic Medicine, Nationwide Children’s Hospital, Columbus, OH, United States of America; 5 EMBL-EBI, Cambridge, United Kingdom; 6 Environmental Genomics and Systems Biology, Lawrence Berkeley National Laboratory, Berkeley, CA, United States of America; 7 Department of Ophthalmology, Klinikum Saarbrücken, Saarbrücken, Germany; 8 Department of Ophthalmology, Saarland University Medical Center, Homburg/Saar, Germany; 9 Department of Biomedical Informatics, University of Colorado Anschutz Medical Campus, Aurora, CO, United States of America; 10 European Genome-Phenome Archive (EGA) in the Centre for Genomic Regulation (CRG), The Barcelona Institute of Science and Technology, Barcelona, Spain; 11 University of Zurich and Swiss Institute of Bioinformatics, Zurich, Switzerland; 12 Institute for Systems Genomics, University of Connecticut, Farmington, CT, United States of America; Brigham Young University, UNITED STATES

## Abstract

The Global Alliance for Genomics and Health (GA4GH) is a standards-setting organization that is developing a suite of coordinated standards for genomics. The GA4GH Phenopacket Schema is a standard for sharing disease and phenotype information that characterizes an individual person or biosample. The Phenopacket Schema is flexible and can represent clinical data for any kind of human disease including rare disease, complex disease, and cancer. It also allows consortia or databases to apply additional constraints to ensure uniform data collection for specific goals. We present phenopacket-tools, an open-source Java library and command-line application for construction, conversion, and validation of phenopackets. Phenopacket-tools simplifies construction of phenopackets by providing concise builders, programmatic shortcuts, and predefined building blocks (ontology classes) for concepts such as anatomical organs, age of onset, biospecimen type, and clinical modifiers. Phenopacket-tools can be used to validate the syntax and semantics of phenopackets as well as to assess adherence to additional user-defined requirements. The documentation includes examples showing how to use the Java library and the command-line tool to create and validate phenopackets. We demonstrate how to create, convert, and validate phenopackets using the library or the command-line application. Source code, API documentation, comprehensive user guide and a tutorial can be found at https://github.com/phenopackets/phenopacket-tools. The library can be installed from the public Maven Central artifact repository and the application is available as a standalone archive. The phenopacket-tools library helps developers implement and standardize the collection and exchange of phenotypic and other clinical data for use in phenotype-driven genomic diagnostics, translational research, and precision medicine applications.

The article "Phenopacket-tools: Building and validating GA4GH Phenopackets" was published in 2023. Journal: PLoS One.

## Introduction

Phenotypic features (signs, symptoms, laboratory and imaging findings, etc.) are of high clinical importance, but standards for recording and exchanging such information along with genomic data have lagged behind. To address this shortfall and pave the way to improving patient care and clinical outcomes, the Global Alliance for Genomics and Health (GA4GH) [1] has developed the Phenopacket Schema, a standard for sharing disease and phenotype information. A phenopacket characterizes an individual person or biosample, linking that individual to phenotypic descriptions, genetic information, diagnoses, and treatments [2].

The Phenopacket Schema enables comparison of sets of phenotypic attributes from individual patients. Such comparisons can aid in diagnosis and facilitate patient classification and stratification for identifying new diseases and treatments [3]. The Phenopacket Schema is designed to support interoperability between the people, organizations, and systems that comprise the worldwide effort to address human disease and biological understanding. These partners include clinical laboratories, authors, journals, clinicians, data repositories, patient registries, electronic health record (EHR) systems, and knowledge bases.

Since its introduction in 2019, the Phenopacket Schema has seen wide adoption. It was recently accepted by the International Standards Organization (ISO) (https://www.iso.org/standard/79991.html). A number of databases and projects have adopted the standard to represent the clinical data of individuals, such as Japan’s biobanking system and the EBI Biosamples repository. An estimated 1 million phenopackets have been created using version 1 of the schema. Increasing the volume of standardized and computable data across a diversity of systems supports global computational disease analysis by integrating genotype, phenotype, and other multi-modal data for precision health applications.

The article "Phenopacket-tools: Building and validating GA4GH Phenopackets" was published in 2023. Journal: PLoS One.

Phenopackets use shared and well-established ontologies, that is, logically defined hierarchies of terms that allow sophisticated algorithmic analysis over medically relevant abnormalities [3]. The Phenopacket Schema does not directly model -omics data in detail but does enable users to link a phenopacket to files representing data from high-throughput screening techniques or to denote individual variants in several formats (see section on VRS and VRSATILE, below) [4]. The Phenopacket Schema integrates a version of the GA4GH Variant Representation Specification and is designed to be interoperable with other GA4GH standards including those for pedigree data.

Previously introduced schemas for clinical data include the Fast Healthcare Interoperable Resources (FHIR) model and the Observational Medical Outcomes Partnership (OMOP) Common Data Model, which are designed for electronic healthcare record (EHR) data, and special-purpose models such as the International Cancer Genome Consortium Accelerating Research in Genomic Oncology (ICGC ARGO) Data Dictionary [5–7]. However, none of these schemas represents a general model for representing clinical data of individual patients with arbitrary diseases and with linkage to genomic and pedigree data.

Phenopackets are designed to be both human- and machine-interpretable, enabling computing operations and validation on the basis of defined relationships between diagnoses, lab measurements, and genotypic information. They also enable seamless transfer of data from a data source (e.g., a document describing the phenotypic information) to a data receiver (e.g., an application that reads and uses it). The Phenopacket Schema aims to provide sufficient and shareable information, including data from EHRs, research studies, data entry tools, published case reports, and other sources to enable capturing of structured clinical data that can be leveraged for computational analysis in other clinical or research environments.

Currently, a wide range of ad hoc database schemas are used to represent clinical data for specific research projects, and numerous different ontologies are used to represent clinical entities; for instance, diseases can be represented by terms from ontologies and terminologies including Mondo, OMIM, Orphanet, NCIt, ICD, and many others [8]. Therefore, the Phenopacket Schema is intentionally flexible in its choice of source ontologies to facilitate wide adoption and to increase the value of the network of systems sharing phenopackets for computational use. The major goals for the Phenopacket Schema include composability, traceability (data provenance), the FAIR principles (Findable, Accessible, Interoperable, and Reusable), and computability [9–12].

The article "Phenopacket-tools: Building and validating GA4GH Phenopackets" was published in 2023. Journal: PLoS One.

Here, we present phenopacket-tools, a software library that makes it easier to create, validate, and work with phenopackets. The library provides a concise builder API to simplify creation of phenopackets in data entry or extract-transform-load pipelines or graphical user interfaces and includes terms from a core set of ontologies to promote interoperability in the community. Additionally, the library provides functionality for converting phenopackets from the v1 data model into the latest v2 format and includes a data validation framework, allowing additional constraints to be enforced for specific use cases. In addition to the API, phenopacket-tools functionality is available through a command-line interface.

## Materials and methods

Phenopacket-tools is a Java library and application for creating, converting and validation of GA4GH Phenopackets. The library is implemented in Java version 17 and takes advantage of Java Platform Module System (JPMS), a feature that promotes modular software architecture and enables deployment of Java applications as efficient runtime images with small binary size. Following the JPMS philosophy, we designed phenopacket-tools as a set of loosely coupled modules, each providing a narrow scope of functionality and depending on a small number of well-maintained external open-source libraries. Note that, although we designed phenopacket-tools as a modular library, the library can still be used in traditional Java class path runtime configurations or from other programming languages that compile to Java byte code such as Kotlin and Scala.

Phenopacket-tools functionality is divided into three categories: *builder* for creating phenopackets using a concise API and promoting a key set of ontologies, *converter* for transforming phenopackets from v1 format to v2 format, and *validator* for checking syntax, semantic constraints, and enforcing project-specific requirements. All of these can be accessed via the API or the command line.

### Brief introduction to protocol buffers

The Phenopacket Schema was created using the open source protocol buffers framework (“protobuf” for short) developed by Google [13]. Protocol buffers provide a language-neutral, platform-neutral, and extensible mechanism for serializing structured data. Protobuf representations can be converted by the protobuf compiler into native bindings for many different computer languages, including Java and Python, thereby providing a widely used framework for working with phenopackets. Additionally, protobuf output can easily be converted into JSON or YAML for human consumption.

The article "Phenopacket-tools: Building and validating GA4GH Phenopackets" was published in 2023. Journal: PLoS One.

Without phenopacket-tools, code for working with phenopackets would need to use the protobuf framework, which generates bindings, i.e., Java class files with definitions of immutable data structures corresponding to the schema elements as well as builder classes for creating hierarchical elements of the Phenopacket Schema. However, the protobuf-generated classes can be verbose and unwieldy. Phenopacket-tools provides terms and constants that are more convenient to use than creating the equivalent terms using the protobuf-generated bindings, and a concise API for creating phenopackets and accessing the ontology concepts from recommended ontologies.

Protobuf uses the term “message” to refer to any hierarchical structure, whereby one message can contain other messages. For instance, an entire phenopacket is a protobuf message and a phenopacket may contain messages that represent other elements such as the PhenotypicFeature and the Measurement. In the following, we will use “message” to refer to a component of the Phenopacket Schema.

### Predefined ontology terms

Currently, numerous different ontologies are used to represent clinical entities. Although the Phenopacket Schema is flexible enough to accept any ontology, it would facilitate interoperability if the community of users of the Phenopacket Schema converged around a set of ontologies that should be used unless there is an application-specific reason for not doing so. For instance, a search in BioPortal [14] for “Unilateral” reveals matches in 36 different ontologies. If users of the Phenopacket Schema chose to use terms representing the concept of unilaterality from 36 different ontologies, then one would need to map the phenopackets post hoc to some common representation, and so on for all the other concepts that are represented in various ontologies. To avoid this Tower of Babel situation, phenopacket-tools encourages the use of a flexible but constrained set of ontology terms from a small number of carefully chosen ontologies (based on computability, currency, open access status, and relevance to genomic health).

### Predefined constants for terms from the core ontologies

Phenopacket-tools provides predefined ontology term constants to enhance interoperability. The library includes a module with the corresponding constant values chosen from a range of areas that can be accessed by calling static functions as shown in Table 1. For example, the Unified Code for Units of Measure (UCUM) provides a simple and widely used syntax to express all common units. In the GA4GH Phenopacket Schema, units are required to report the results of laboratory tests (*Measurement* message) and to specify the dosage of medication and some other treatments (*MedicalAction* message). In the GA4GH Phenopacket Schema, units are represented as OntologyClass messages and we recommend UCUM for representing units. For instance, milligram is UCUM:mg, microgram per deciliter is UCUM:ug/dL, and millimeters of mercury (used to specify blood pressure) is UCUM:mm[Hg]. The corresponding static function names in phenopacket-tools are Unit.milligram(), Unit.microgramPerDeciliter(), and Unit.mmHg().

The article "Phenopacket-tools: Building and validating GA4GH Phenopackets" was published in 2023. Journal: PLoS One.

**Table 1:** Utility classes in the org.phenopackets.phenopackettools.builder.builders package that provide predefined constants that simplify construction of selected elements of the Phenopacket Schema. The second column shows an example, and a full list is available in the online documentation. The third column indicates the parts of the Phenopacket Schema in which the constants can be used.

Class	Static function	Phenopacket element	Source ontology or terminology
Unit	mmHg()	Measurement, MedicalAction	UCUM
Severity	mild()	PhenotypicFeature	HPO
Laterality	unilateral()	PhenotypicFeature	HPO
SpatialPattern	perilobular()	PhenotypicFeature	HPO
Evidence	selfReportedPatientStatementEvidence()	PhenotypicFeature	ECO
Gender	identifiesAsMale()	Individual	LOINC
BiospecimenType	bloodDNA()	Biosample	NCIT
PathologicalTnm	pM1StageFinding()	Biosample	NCIT
MaterialSample	referenceSample()	Biosample	EFO
AllelicState	heterozygous()	Interpretation	GENO
DiseaseStage	nyhaClassIII()	Disease	NCIT
Organ	kidney()	Disease	UBERON
Response	partialRemission()	MedicalAction	NCIT
AdministrationRoute	intravenous()	MedicalAction	NCIT

For representing the evidence of assertions, terms from the Evidence and Conclusion Ontology (ECO) should be used where possible [15]. For phenopackets derived by manual annotation of a published case report, the constant Evidence.authorStatementFromPublishedClinicalStudyManualAssertion() should be used. For automatic generation of phenopackets from published reports (e.g., by text mining), Evidence.authorStatementFromPublishedClinicalStudyAutomaticAssertion() should be used. Given the wide range of evidence available for clinical data, terms from other ontologies may be used where appropriate.

Terms from the National Cancer Institute’s Thesaurus (NCIt) are used to represent a number of different subject areas [16]. Clinical Modifier and Onset terms are taken from the Human Phenotype Ontology (HPO) [17]. Finally, two terms from the Experimental Factor Ontology (EFO) are used to represent disease and reference sample status.

The article "Phenopacket-tools: Building and validating GA4GH Phenopackets" was published in 2023. Journal: PLoS One.

We do not have recommendations for concepts that are not discussed here, and users should choose application-specific terminologies or ontologies based on their needs and the criteria mentioned earlier.

### Convenience functions

The phenopacket-tools library provides several convenience functions to reduce the amount of boilerplate in client code (in this context, client refers to application-specific code developed by a user of the phenopacket-tools library which calls the methods provided by the library).

The *OntologyClass* message is used ubiquitously in the Phenopacket Schema. Each *OntologyClass* message has two fields, id (e.g., “HP:0001250”) and label (e.g., Seizure). Using the Builder provided by the protobuf framework requires four commands to be chained (Fig 1A). The phenopacket-tools library provides predefined constants accessible via static functions for commonly used ontology classes that will be discussed in the next section (an example is shown in Fig 1B). In addition, a convenience function can be used to generate an arbitrary ontology class (Fig 1C) to reduce the verbosity of client code. All three code snippets produce the identical output (Fig 1D). Analogous functions are provided for many other areas (Table 2).

**Fig 1:** Methods for creating OntologyClass messages with phenopacket-tools. A. Builder pattern provided by the protobuf Java framework. B. Predefined constant (static function) that returns an Ontology term singleton instance. Here, BiospecimenType.bloodDNA() generates the ontology term that represents the NCI Thesaurus (NCIt) concept C158416 for the biospecimen type “blood DNA” C. Convenience function provided by phenopacket-tools. D. The JSON representation of *OntologyClass* message that is generated by the code in panels A, B, and C.

**Table 2:** Examples of convenience functions. In addition to the ontologyClass function that was explained in detail in the text, phenopacket-tools provides convenience functions to reduce the amount of boilerplate in client code. Details are available in the online user guide and Javadoc documentation.

Class	Function
OntologyClass	ontologyClass(String id, String label)
Age	age(String iso8601duration)
Expression	hgvsCdna(String hgvsExpression)
Extension	alleleFrequency(double frequency)
Resource	hpoVersion(String version)
TimeElement	gestationalAge(int weeks, int days)
TimeElement	childhoodOnset()

### Concise builders

The API of the phenopacket-tools library simplifies the construction of the various components of the Phenopacket Schema with concise builders that wrap the code generated by the protobuf compiler into convenience functions and an API to guide creation of valid Phenopacket elements, reduce verbosity, and increase code legibility. The org.phenopackets.phenopackettools.builder package provides a builder class for each Phenopacket element. We designed the builders such that all required fields must be provided upon builder creation, to prevent generation of invalid elements. Each element can be further customized by chaining additional functions to the builder methods to specify optional components of the message such as an enumerated attribute value (e.g., a variant actionability class) or a custom value as a component’s attribute. For instance, to create a *PhenotypicFeatureBuilder*, an *OntologyClass* corresponding to the *type*, a required attribute of a *PhenotypicFeature*, must be provided to instantiate the builder. The builder further offers convenience methods for setting the optional *PhenotypicFeature* attributes, either as predefined constants such as builder.childhoodOnset() or custom values such as builder.iso8601onset("P10Y4M2D"). The building process is concluded by calling build(), yielding the final element. The phenopacket-tools builder code is typically substantially less verbose than the equivalent protobuf-generated builder code, providing a concise and intuitive interface. The builders can be used in conjunction with the predefined constants and convenience functions that were explained in the previous sections (Fig 1).

The article "Phenopacket-tools: Building and validating GA4GH Phenopackets" was published in 2023. Journal: PLoS One.

Below, we briefly discuss how some of the key elements (messages) in the Phenopacket Schema are supported by phenopacket-tools builder methods.

### Individual

Each phenopacket describes one individual. In many cases, the individual is a patient or a proband of a study. The *Individual* message specifies demographic information. For example, enumerations are used to represent biological sex (MALE, FEMALE, OTHER, UNKNOWN) and chromosomal sex (XY, XX, XO, XXY, XXX, XXYY, XXXY, XXXX, XYY, OTHER, UNKNOWN). The *Individual* element additionally has an optional field for gender. Phenopacket-tools provides LOINC (Logical Observation Identifiers Names and Codes) codes to represent gender, for instance, *Female-to-male transsexual* (LOINC:LA22880-1), corresponding to the static function Gender.femaleToMaleTranssexual().

### Phenotypic feature

A *PhenotypicFeature* message describes clinical abnormalities including signs and symptoms, laboratory findings, imaging, and electrophysiological results, along with modifier and qualifier concepts. Each phenotypic feature should be described using a term from the Human Phenotype Ontology (HPO), a rich representation of abnormal human phenotypic features. The HPO is complemented by a corpus of phenotype annotations (HPOA) corresponding to each of over 8,400 rare diseases [17, 18]. Almost all clinical genetics diagnostic tools now leverage the HPO to encode and compute over patient features in the context of genomic variant classification. Accurate and comprehensive phenotyping matters for accurate diagnosis. Many exome and genome sequencing pipelines incorporate phenotype analysis into approaches for ranking and interpreting variants [19].

The article "Phenopacket-tools: Building and validating GA4GH Phenopackets" was published in 2023. Journal: PLoS One.

The *PhenotypicFeature* has optional fields that can be used to provide context about a phenotypic abnormality. The severity field is used to describe the intensity or degree of the phenotypic feature. The HPO defines five relevant terms (Borderline, Mild, Moderate, Severe, Profound), each of which has a corresponding static function such as Severity.mild().

The modifiers field can contain a list of terms that describe the frequency, laterality, or another pattern of a certain phenotypic feature in the patient being described. We recommend using terms from the Clinical Modifier subontology of the HPO. There are over 250 available terms, and we provide constants for some commonly used terms for laterality, e.g., Laterality.unilateral(), and spatial pattern, e.g., SpatialPattern.perilobular().

### Measurement

The *Measurement* message is used to capture quantitative, ordinal (e.g., absent/present), or categorical measurements. LOINC assigns a unique identifier to a fixed combination of six parts: Component (the measured analyte), Property (measured quantity of the analyte, e.g., mass), Time Aspect (moment in time or a time interval, e.g., 24-h urine), System (sample material, e.g., serum), Scale (level of measurement e.g., quantitative), and Method [20]. We recommend using LOINC codes to denote the assay of *Measurement* messages.

### Biosample

A *Biosample* message encodes information about the examination of biological specimens such as tissue biopsies. One example use case would be to describe the biopsy of a tumor and of surrounding normal tissue. Another example would be to describe a muscle biopsy in a patient with muscular dystrophy. Some of the fields of the biosample are cancer-specific, but because these fields are optional, the *Biosample* message can be used to describe any kind of biological specimen.

The National Cancer Institute (NCI) Thesaurus (NCIt) provides a reference terminology with over 100,000 terms and textual definitions. Although the focus is on cancer, terms from many other domains are included [16]. We recommend that NCIt terms be used to describe cancers and related data types such as cancer staging, cancer biomarkers, and procedures. The term field of the top-level *PhenotypicFeature* messages should be created with HPO terms. In contrast, the *PhenotypicFeature* message in the *Biosample* is meant to refer to the phenotypic features of a biopsy or similar biospecimen. Terms from the NCIt can be used to refer to cancer-related features. If the *Biosample* refers to a specimen that is not cancer-related, for instance a muscle biopsy obtained from a person with muscular dystrophy, then HPO terms can be used. The *Measurement* field should be created as described above but is used to describe phenotypic features or measurements of the biospecimen.

The article "Phenopacket-tools: Building and validating GA4GH Phenopackets" was published in 2023. Journal: PLoS One.

The *sampled_tissue* field of the Biosample denotes the tissue from which a biopsy or other tissue specimen was obtained. Uberon is an integrated cross-species ontology consisting of over 21,000 classes representing a variety of anatomical entities, organized according to traditional anatomical classification criteria [21]. Uberon should be used to specify organs and other anatomic entities, for instance, to represent the body site at which a biosample was taken. Phenopacket-tools provides predefined UBERON classes representing commonly used anatomical entities such as eye or kidney. In clinical use, it is most common to denote the site of tumor origin with International Classification of Diseases for Oncology (ICD-O) Topography (T), together with the ICD-O Morphology (M) code which indicates histological type and degree of malignancy. Tools such as *icdot2uberon* can be used to convert between ICD codes and UBERON classes [22].

The *sample_type* field denotes the kind of specimen (DNA, RNA, protein, histology, etc.) that is derived from the sampled tissue. The specimen type should be specified using terms that descend from the NCIt term for *Biospecimen* (NCIT:C70699). Phenopacket-tools provides a number of constants for many of these terms, e.g., BiospecimenType.bloodDNA().

Staging of cancer expresses the extent that cancer has spread and is usually described by numbers I to IV with IV representing distant extension beyond the organ of origin, diffuse infiltration or metastatic spread. Clinical stage is based on all of the available information obtained before a surgery to remove the tumor, while pathologic stage adds additional information gained by examination of the tumor microscopically after surgery and refers to the stage before therapy. If desired, clinical stage can be expressed in the *Disease* message using the disease_stage or clinical_tnm_finding fields. The *pathological_stage* field, which is used in *Biospecimen*, should be used with terms such as *Lung Cancer by AJCC v8 Stage* (NCIT:C136467) from the NCIt.

The *pathological_tnm_finding* field is used to represent TNM findings used to determine the pathological stage. Staging is often based on the TNM system, involving the tumor size (T) and the regional lymph node involvement (N) and/or distant metastasis (M). Again, we recommend using NCIt terms for this field. Predefined terms are provided for general TNM findings (note that some cancers have bespoke TNM classifications that are not provided here). For instance, PathologicalTnm.pM1StageFinding() refers to pathological stage M1 (distant spread of cancer, i.e., metastasis).

The article "Phenopacket-tools: Building and validating GA4GH Phenopackets" was published in 2023. Journal: PLoS One.

The *material_sample* element of the *Biosample* message can be used to specify the status of the sample. For instance, a sample may be used as a normal control, often in combination with another sample that is thought to contain a pathological finding. We recommend terms from the Experimental Factor Ontology (EFO) subclasses of *Material Sample* (OBI:0000747), e.g., *abnormal sample* (EFO:0009655).

### Interpretation

A phenopacket can contain one or more *Interpretation* elements that specify interpretations of genomic findings. We refer to the online documentation and to our detailed introduction [23] for further details. We provide constants for one field that is used in the *Interpretation*.

The *allelic_state* element should use terms from the GENO ontology to specify the allelic state (zygosity). Static functions are provided for *homozygous* (GENO:0000134), *heterozygous* (GENO:0000135), and *hemizygous* (GENO:0000134).

Genomic variants can be encoded in the GA4GH Variation Representation Specification (VRS) format. When introduced in Phenopackets v2, a protobuf version of VRS (github.com/ga4gh/vrs-protobuf) was derived from the source VRS representation in JSON schema and used for Phenopackets. In Phenopackets-tools, we translate this derived representation back to JSON schema, resulting in a message structure that is losslessly transformable but syntactically distinct from the native VRS JSON schema. For users that wish to express Phenopackets with a native VRS representation, we have implemented a function that converts VRS objects in Phenopackets into JSON objects that correspond to the native VRS schema. If users desire to interact with databases or software that use the VRS schema, this function can be used to generate conformant JSON code.

### Disease

The term element of Disease is used for an ontology term that specifies a disease. Phenopackets can contain a list of Disease messages that represent diseases diagnosed in the proband. To represent diseases, we recommend the Mondo Disease Ontology which integrates and harmonizes multiple disease terminologies and ontologies into a coherent logic-based ontology that provides precise semantic mappings between terms. Mondo aims to systematically integrate the classifications and relationships in partnering terminological resources into a semantically coherent, single resource to enable the aggregation and analysis of disparate clinical data repositories and facilitate the discovery of relationships between disease concepts across systems. Mondo terms include links to many other nosologies and disease ontologies [24]. Some users may prefer OMIM, ORDO, or NCIt terms, but since Mondo imports and provides provenance and attribution to these source ontologies, it is nearly always possible to use Mondo.

The article "Phenopacket-tools: Building and validating GA4GH Phenopackets" was published in 2023. Journal: PLoS One.

The *disease_stage* field can be used to represent the disease stage according to the appropriate disease-specific clinical staging systems. As an example, we provide predefined classes for cancer Stage 0-Stage IV and New York Heart Association stages for heart failure, e.g., DiseaseStage.nyhaClassIII().

The *clinical_tnm_finding* field should be used to represent clinical tumor/node/metastasis cancer-related findings using terms from the NCIt.

The *primary_site* field is used to specify the organ primarily affected by the disease. Uberon should be used to specify organs and other anatomic entities. The *laterality* field should use HPO constants for laterality (Table 1).

*MedicalAction*. The MedicalAction message can represent four specific kinds of medical action: *Procedure*, *Treatment*, *RadiationTherapy*, and *TherapeuticRegimen*. In some cases, terms from the Medical Action Ontology (MAxO) can be used. MAxO is an ontology of medical interventions including therapy and other actions for clinical management. The current focus of MAxO is on rare disease but terms are available for all classes of disease. MAxO is available at https://github.com/monarch-initiative/MAxO and can be viewed in the Ontology Lookup Service of the European Bioinformatics Institute, BioPortal, and OntoBee [14, 25, 26]. We recommend that where possible MAxO terms be used for the *MedicalAction* message of the GA4GH Phenopacket Schema.

For *Procedure*, the *code* field should use Terms from either MAxO or NCIt and the *body_site* field should use Uberon terms to specify organs and other anatomic entities.

For *Treatment*, the *agent* field represents a compound or other agent administered to a patient. Numerous resources are available for specifying pharmaceutical compounds, drug names, and related data. RxNorm is a standard and freely available terminology maintained by the U.S. National Library of Medicine (NLM) that includes normalized names and relationships extracted from several proprietary drug knowledge bases [27]. RxNorm can be interrogated through the RxNav browser, or via APIs (https://lhncbc.nlm.nih.gov/RxNav/). DrugBank is a web-enabled database containing comprehensive molecular information about drugs, their mechanisms, their interactions, and their targets [28]. DrugBank content on the platform is provided under, and subject to, a Creative Commons Attribution-NonCommercial 4.0 International License but there are some restrictions on commercial use. DrugCentral (freely available via CC-BY-SA) integrates a broad spectrum of drug resources related to chemical structures, biological activities, regulatory data, pharmacology, disease information, and drug formulations [29]. DrugCentral associates clinical data with drugs in two distinct ways: medical uses and adverse events. Disease terms, mapped to SNOMED_ID and DO_ID where possible, are available for indications and off-label drug uses, as well as contra-indications. All drug-related adverse events in DrugCentral are mapped to the MedDRA (Medical Dictionary for Regulatory Activities, https://www.meddra.org/) terminology. Adverse events are sorted by importance (specifically, the log likelihood ratio [30]) and separately provided for women, men, elderly people, and children, where data is available. All drug pharmacologic actions are captured in DrugCentral and mapped to ATC (Anatomic Therapeutic and Chemical Classification system, https://www.whocc.no/), ChEBI (Chemical Entities of Biological Interest [31]), and MeSH, where available. Side effects, separated by sex, are also mapped in DrugCentral. ChEMBL is a manually curated database of bioactive molecules with drug-like properties. It brings together chemical, bioactivity and genomic data to aid the translation of genomic information into effective new drugs [32]. We recommend that one of these resources be used according to project needs.

The article "Phenopacket-tools: Building and validating GA4GH Phenopackets" was published in 2023. Journal: PLoS One.

For *Treatment*, the *route_of_administration* field represents the part of the body or way a drug is administered, e.g., by mouth or intravenously. Terms that descend from the NCIt term Route of Administration (NCIT:C38114) should be used. The phenopacket-tools library provides constants for many of these terms, e.g., AdministrationRoute.intravenous() (Table 1). The *intent* field represents the condition or disease that this treatment was intended to address. In general, the disease should be listed in the Diseases section and the same ontology term should be used.

Finally, the MedicalAction has several fields that can be used with any of the four kinds of medical action. The *response_to_treatment* field is intended for concepts such as *Partial Remission* (NCIT:C18058) from the NCI Thesaurus that can be used to code the overall response of a patient to treatment. Predefined ontology terms are available (Table 1). The *adverse_events* field is a list of adverse effects experienced by the patient attributed to the treatment. Terms from the HPO or the Ontology of Adverse Events [33] can be used. The *treatment_termination_reason* field is used to represent the reason for stopping a medical action. The phenopacket-tools library provides several concepts from the NCIT that describe the reason for which a treatment was stopped, such as *Treatment Completed as Prescribed* (NCIT:C105740) and *Treatment Terminated Due to Toxicity* (NCIT:C105741).

### Convert phenopackets from v1 to v2

Phenopacket-tools provides a method for mapping Phenopacket Schema from v1 to v2 data model. The mapping functionality is offered in the Java API as *V1ToV2Converter* and in the *convert* command of the command-line interface. The conversion is lossy due to the breaking changes made to the *Variant* element of the v1 schema, and extra care must be taken when converting data that include this element. To prevent unintended results, the conversion of *Variant* elements is disabled by default in the command-line tool. However, the *Variant* element can be converted if the v1 data includes exactly one *Disease* and the disease can be assumed to be the definitive diagnosis. If this is the case, then each variant is converted into *VariantInterpretation* and assumed to be causative of the diagnosis. The variant interpretation must contain American College of Medical Genetics and Genomics (ACMG) variant pathogenicity and a therapeutic actionability to meet the validation requirements. Since this information is absent in the v1 data model, the variant is assigned “not provided” ACMG variant pathogenicity and “unknown” therapeutic actionability. However, the phenopacket-tools API code can be used as the basis of custom conversion logic that reflects assumptions of the original dataset.

### Validate phenopackets

The Phenopacket Schema uses the protobuf framework to define the structure of the schema components and the hierarchical arrangement of the components. However, the framework does not provide any means to validate content apart from basic checks that, for instance, a field contains a number, string, or another message (hierarchical component). Any additional validation is delegated to downstream applications. Phenopacket-tools provides an extensible API for validation of all schema components, including a model of validation workflow and validation results.

The validation workflow consists of a list of steps. The workflow includes a mandatory *base* validation step that validates syntax and cardinality of each component, to verify the basic requirements of the Phenopacket Schema, such as presence of identifier fields and metadata (see the online documentation). The base validation is implemented using JSON schema. The workflow can be extended by any number of validation steps for checking specific logical or semantic requirements. Phenopacket-tools offers an API for the validation steps to allow encoding custom validation logic as well as several off-the-shelf validators.

The article "Phenopacket-tools: Building and validating GA4GH Phenopackets" was published in 2023. Journal: PLoS One.

The central element of the validation API is *PhenopacketValidator* that represents a single validation step. The validator is identified by *ValidationInfo* with the name, type, and description of the validation functionality. The validation reports any errors as *ValidationResult* objects, one result per error. The execution of the workflow is orchestrated by the *ValidationWorkflowRunner*. The runner applies the validators in the correct order, ensuring that the base validator is applied as first, and gathers the results into a *ValidationResults* container. The container represents the results of the validation as immutable value objects, *ValidatorInfo*, *ValidationResult*, suitable for reporting back to the user.

Phenopacket-tools provides off-the-shelf validators for common checks. The metadata validator verifies presence of a *Resource* element for any ontology concept to ensure unambiguous concept resolution. The ancestry validator checks violations of the annotation propagation rule; the phenopacket must not contain both term and its ancestor. The only exception is presence of an observed ancestor and an excluded child (e.g. observed *Abnormality of finger* and excluded *Arachnodactyly*). The organ system validator uses HPO to check if phenopacket includes phenotypic feature for selected organ systems represented by a top-level HPO term. Finally, a custom JSON schema can be used to enforce presence and format of Phenopacket Schema components (Table 3). The validators can be used by calling the appropriate API methods from the client code or from the command line.

**Table 3:** An overview of validation errors. Phenopacket-tools includes multiple off-the-shelf validators for performing basic and domain-specific checks. The validators emit errors that refer to invalid phenopacket components. The table lists the errors and solutions for issues discovered in example phenopackets that are included in the phenopacket-tools distribution.

Example phenopacket	Validator	Validation error	Solution
missing-fields	BaseValidator	‘id’ is missing but it is required	Add the phenopacket ID
missing-fields	BaseValidator	‘subject.id’ is missing but it is required	Add the subject ID
missing-fields	BaseValidator	‘phenotypicFeatures[0].type.label’ is missing but it is required	Add the label attribute into the type of the first phenotypic feature
missing-resources	MetaDataValidator	No ontology corresponding to ID ‘NCBITaxon:9606’ found in MetaData	Add a *Resource* element with NCBITaxon definition into *MetaData*
marfan.no-subject	CustomJsonSchemaValidator	‘Subject’ is missing but it is required	Add the *Subject* (*Individual* message)
marfan.no-phenotype	CustomJsonSchemaValidator	‘phenotypicFeatures’ is missing but it is required	Add at least one *PhenotypicFeature*
marfan.not-hpo	CustomJsonSchemaValidator	‘phenotypicFeatures[0].type.id’ does not match the regex pattern ^HP:\d{7}$	Use HPO in the type.id of the first phenotypic feature
marfan.no-time-at-last-encounter	CustomJsonSchemaValidator	‘subject.timeAtLastEncounter’ is missing but it is required	Add the time at last encounter
marfan.obsolete-term	HpoPhenotypeValidator	Using obsolete id (HP:0002631) instead of current primary id (HP:0002616) in id-C	Replace the obsolete ID with the primary ID
marfan.annotation-propagation-rule	HpoAncestryValidator	Phenotypic features of id-C must not contain both an observed term (Aortic root aneurysm, HP:0002616) and an observed ancestor (Aortic aneurysm, HP:0004942)	Remove the ancestor term
marfan.missing-eye-annotation	HpoOrganSystemValidator	Missing annotation for Abnormality of the eye [HP:0000478] in id-C	Annotate the eye or exclude any abnormality

The article "Phenopacket-tools: Building and validating GA4GH Phenopackets" was published in 2023. Journal: PLoS One.

## Results and discussion

### Code availability

Phenopacket-tools is open source, and is available on GitHub under the GNU3 license. We follow the semantic versioning system [34] to tag and release our library. The version described in this paper is v1.0.0. Releases are published on the Maven Central repository to allow users to use the phenopacket-tools library in their applications. Comprehensive API documentation, a user guide, and a tutorial are available on http://phenopackets.org/phenopacket-tools. A prebuilt executable Java archive with the command-line interface for the end users is available for download from GitHub releases section. Alternatively, the application can be built with a single command on Windows (mvnw.cmd package), or on macOS or Linux (./mvnw package).

### Usage examples

In this section, we outline common procedures that involve working with GA4GH Phenopacket data. When working with existing phenopacket files, we use PhenopacketParser and PhenopacketPrinter from the phenopacket-tools-io module for (de)serialization of phenopacket, family, or cohort from/to protobuf binary, JSON or YAML data formats.

### Building phenopackets

Although Java bindings generated by the protobuf compiler can be used to work with phenopackets, the bindings are not easy to use. Phenopacket-tools simplifies the process of reading or writing phenopackets by providing static functions to generate commonly used elements such as left(), convenience functions, and concise builders (Methods). The protobuf version and the corresponding phenopacket-tools version as well as the generated JSON code (Figs 1 and 2).

The article "Phenopacket-tools: Building and validating GA4GH Phenopackets" was published in 2023. Journal: PLoS One.

**Fig 2:** Building phenopackets. Phenopacket-tools offers convenience functions that streamline the construction of GA4GH phenopackets. (A) The protobuf framework automatically generates Java bindings for messages that are defined in proto files. This panel shows an example of how the bindings can be used to create a *PhenotypicFeature* element that represents severe weakness of the left triceps muscle with age of onset at eleven years and four months (“P11Y4M”). (B) Phenopacket-tools provides builder classes that contain convenience functions that hide the relative verbosity of the protobuf bindings. (C) JSON representation of the *PhenotypicFeature* element generated by Panel A or B.

Several examples of how to use the library to create phenopackets are provided in the source code of the command-line interface module of the library. We anticipate that the library code will be used as a part of applications that leverage user-entered data or transform data from other sources to generate phenopackets rather than building phenopackets for specific cases as we have done here. However, the examples demonstrate numerous common use cases and can be extended for many purposes in application code.

### Converting phenopackets

Version 1 of the GA4GH Phenopacket Schema was released in 2019 to elicit community feedback. In response to this feedback, the schema was extended and refined and version 2 was released in 2021 and published in 2022 by the International Standards Organization (ISO) as ISO 4454:2022 [35]. The representation of versions 1 and 2 of the *PhenotypicFeature*, which models and contextualizes phenotypic observations, is nearly identical and version 1 phenopackets that contain phenotypic information can be automatically converted to version 2 phenopackets.

The ability to convert between versions 1 and 2 of phenopackets is quite useful, given that over a million phenopackets have been created so far. To demonstrate the conversion functionality, we will use a cohort of 384 probands diagnosed with a Mendelian disease that was used to benchmark the performance of LIRICAL [36] and Exomiser [37], tools for phenotype-driven prioritization of genomic variants and diseases. The probands were represented as v1 phenopackets, including phenotypic features, the causal genomic variants, and the diagnosed disease. To further investigate this dataset, the phenopacket-tools conversion functionality should be used to convert the v1 phenopackets into the current v2 format.

The article "Phenopacket-tools: Building and validating GA4GH Phenopackets" was published in 2023. Journal: PLoS One.

First, a converter (V1ToV2Converter)is obtained from the convert module. The optional conversion of the Variant element of the v1 schema is controlled by a flag in the converter’s constructor. Next, phenopacket JSON files are read into protobuf messages using phenopacket parser (*PhenopacketParser*). The converter maps each message into a v2 phenopacket. The converted phenopackets can be stored to disk using the phenopacket printer (PhenopacketPrinter).

### Validating phenopackets

In protobuf (version 3, which is what the Phenopacket Schema uses), all fields are optional. However, the Phenopacket Schema defines certain fields to be required. Phenopacket-tools uses JSON schema to encode these requirements. Additionally, it may be desirable to enforce additional constraints or requirements on phenopackets that are created for a specific purpose. For instance, one may want to require that phenopackets made for rare-disease diagnostics include the age of the proband and use HPO terms to represent phenotypic features. Additionally, one may want to enforce requirements that are difficult to encode using JSON schema, such as that only a valid term id is used (currently, the HPO has over 16,000 terms), or that the phenopacket does not encode both a term and a parent or ancestor of the term, or that the phenopacket annotates or excludes abnormality in selected organ systems. Here we show a validation workflow for checking all these requirements.

We start by getting a workflow builder (JsonSchemaValidationWorkflowRunnerBuilderxya). The builder automatically adds the base validation backed by a JSON schema and the metadata validator (MetaDataValidator) to check the presence of a *Resource* for the ontology concepts into the workflow. We provide an example of a JSON schema engineered to validate the presence of the age of the proband in a phenopacket. To use the schema in the validation, we set a schema url to the workflow builder (builder.addJsonSchema(customSchema)). We use ontology-dependent validators to point out usage of obsolete HPO term ids (HpoPhenotypeValidators.Primary) and to report violations of the ontology annotation propagation rule (HpoAncestryValidators.Ancestry). Last, we add a validator for checking annotation of selected organ systems (e.g., the cardiovascular system, HpoAncestryValidators.OrganSystem). The validation workflow can be used to validate phenopackets, producing a *ValidationResults* container for each phenopacket (Fig 3). We provide further examples on how to use the interfaces of the phenopacket-tools library to create project-specific validators in the online documentation.

The article "Phenopacket-tools: Building and validating GA4GH Phenopackets" was published in 2023. Journal: PLoS One.

**Fig 3:** Creating a customized validator and applying it to a phenopacket. The ValidationResult object contains fields representing validation metadata, the level of the validation (error or warning), the category, and a message (See Table 3).

### Command-line interface

The command-line interface application allows users to generate phenopacket example files, convert, and validate phenopackets without writing Java code. We designed the CLI application around principles of UNIX philosophy. The commands of the CLI application perform simple and focused tasks and the application supports reading and writing phenopackets from/to standard streams, to allow combining commands into data pipelines. The application reads phenopackets formatted in JSON and YAML data formats and can detect the input data format automatically. For maximizing the user convenience, the application supports command-line autocomplete, showing subcommands, available options and parameters, and a granular adjustment of logging verbosity to facilitate debugging. The source code of the application is designed as a separate module within the phenopacket-tools library and exemplifies usage of the library functionality, serving as an important part of the library documentation.

The GA4GH Phenopacket Schema is designed for sharing disease and phenotype information that characterizes an individual person, linking that individual to detailed phenotypic descriptions, genetic and genomic information, diagnoses, variant interpretations, and treatments. In addition to functioning as a data exchange schema, phenopackets represent computational models of the health trajectory of an individual and can model data from many domains including phenotypic abnormalities, numerical measurements, disease diagnoses, and treatments, optionally linked to genomic functional or variant data [2]. We have previously published a tutorial and detailed example representing a child with retinoblastoma [23]. The Phenopacket Schema is designed to complement and be interoperable with existing schemas for health care and translational research. The Fast Health Interoperability Resources (FHIR) Standard was introduced in 2011 by Health Level Seven International (HL7) and leverages Web technologies such as a Representational State Transfer (REST)-based application programming interface (API), XML, and JSON. Information is represented using building blocks (FHIR resources) that define the content and structure of information and serve as an extensible foundation providing resources, APIs, and a platform in which different solutions can be implemented [38]. The information contained in a phenopacket can be represented in FHIR, and we are currently developing a FHIR Implementation Guide to represent the GA4GH Phenopacket Schema using and extending FHIR resources [39]. The Clinical Data Interchange Standards Consortium (CDISC) Operational Data Standard is dedicated to the exchange of data within clinical trials [40], but is not a general schema for representing comprehensive clinical and genomic data about an individual. However, it may be possible in the future for CDISC to be able to represent collections of Phenopackets in the context of trial data exchange. The Observational Health Data Sciences and Informatics (OHDSI) Observational Medical Outcomes Partnership (OMOP) common data model is frequently used in clinical data warehouses as a foundation for observational research. OMOP enables large-scale analysis of distributed data to generate evidence for research that promotes better health decisions and better care [41]. The Phenopacket Schema is more narrowly focused towards semantic analysis of individual patient disease trajectories, but is compatible with the OMOP Schema; a preliminary transformation strategy from OMOP to GA4GH Phenopacket Schema has been published [42]. Phenopackets are a schema that can and should be used with ontologies and commonly used clinical terminologies such as the Systematized Nomenclature of Medicine Clinical Terms (SNOMED CT) and Logical Observation Identifiers, Names, and Codes (LOINC). We envision the role of the GA4GH Phenopacket as a common exchange format that can improve interoperability between research data and existing clinical systems at the case-level, and the schema is especially well suited to providing a comprehensive and computable representation of clinical data for genomic research and care.

The article "Phenopacket-tools: Building and validating GA4GH Phenopackets" was published in 2023. Journal: PLoS One.

The main motivation for the phenopacket-tools library is the fact that the Java bindings generated by the protobuf framework are not easy to use and do not enforce the constraints defined by the GA4GH Phenopacket Schema. Also, we envision that consortia and project groups using phenopackets will want to define requirements and constraints that go beyond those defined by the schema itself. The library is designed to be used in different settings. Developers of pipelines for genotype-phenotype analysis can use the library to test the validity of input data. Developers of graphical user interfaces for the entry of clinical data can use the library to build code that will generate valid phenopackets. Bioinformaticians developing analysis algorithms for clustering or clinical decision support using data encoded as phenopackets can use the command line tool or the library to perform various processing steps.

As mentioned in the introduction, the GA4GH Phenopacket Schema does not enforce the use of any specific ontology or terminology. Nevertheless, it will promote interoperability if users of the schema employ the same ontologies wherever possible. Therefore, phenopacket-tools provides constants that represent ontology terms for commonly used concepts (Table 1). We prefer open-source ontologies such as those from OBO Foundry wherever possible. However, users are free to use other ontologies or terminologies such as SNOMED CT if these better fit with their analysis goals.

The GA4GH Phenopacket Schema places only a few constraints on the schema elements to facilitate wide adoption in a variety of settings. Consequently, the broadest validation scope that is applicable to all phenopackets is limited to checking the syntax and cardinality of the schema elements, and to ensuring that all ontology concepts can be traced to a specific ontology version. For specific projects, users can design additional constraints to meet the project requirements. Phenopacket-tools provides off-the-shelf validators for performing basic syntax and cardinality checks, including user-specific requirements encoded in JSON schema documents, and sets up the validation framework for building project-specific validators. The library provides an example by implementing validators for checking logical consistency of clinical phenotype data encoded using Human Phenotype Ontology, designed for phenotype-driven diagnostics of Mendelian diseases. The validation framework is open to future improvements. Possible non-trivial extensions include validation of ontology concepts across all phenopacket elements such as medical actions and diagnoses, validation of the longitudinal aspect of the phenotypic annotations, and validation of variation descriptors.

## Conclusion

The GA4GH Phenopacket Schema is designed to support comprehensive and accurate computational analysis of clinical data for research and ultimately clinical decision support. Ontologies are systematic formal representations of knowledge that can be used to integrate and analyze large amounts of heterogeneous data by defining entities and concepts such as genetic variation, clinical findings, and diseases as well as the relationships between these concepts in a way that allows computational logical reasoning [3]. Ontology-driven algorithms have been transformative for rare disease diagnosis [37, 43]. While existing algorithms have leveraged unordered sets of HPO terms to support diagnostics in rare disease, the GA4GH Phenopacket Schema offers the ability to go beyond this by integrating information about the time course of disease manifestations, treatments and other clinical management, quantitative measures, and multimorbidity. We anticipate that phenopacket-tools will help users to leverage the full advantages of this new schema.

The article "Phenopacket-tools: Building and validating GA4GH Phenopackets" was published in 2023. Journal: PLoS One.

## References

[1] RehmHL, PageAJH, SmithL, AdamsJB, AlterovitzG, BabbLJ, et al. GA4GH: International policies and standards for data sharing across genomic research and healthcare. Cell Genom. 2021;1. doi: 10.1016/j.xgen.2021.100029 35072136PMC8774288

[2] JacobsenJOB, BaudisM, BaynamGS, BeckmannJS, BeltranS, BuskeOJ, et al. The GA4GH Phenopacket schema defines a computable representation of clinical data. Nat Biotechnol. 2022;40: 817–820. doi: 10.1038/s41587-022-01357-4 35705716PMC9363006

[3] HaendelMA, ChuteCG, RobinsonPN. Classification, Ontology, and Precision Medicine. N Engl J Med. 2018;379: 1452–1462. doi: 10.1056/NEJMra1615014 30304648PMC6503847

[4] den DunnenJT. Describing Sequence Variants Using HGVS Nomenclature. Methods Mol Biol. 2017;1492: 243–251. doi: 10.1007/978-1-4939-6442-0_17 27822869

[5] Bender D, Sartipi K. HL7 FHIR: An Agile and RESTful approach to healthcare information exchange. Proceedings of the 26th IEEE International Symposium on Computer-Based Medical Systems. 2013. pp. 326–331.

[6] VossEA, MakadiaR, MatchoA, MaQ, KnollC, SchuemieM, et al. Feasibility and utility of applications of the common data model to multiple, disparate observational health databases. J Am Med Inform Assoc. 2015;22: 553–564. doi: 10.1093/jamia/ocu023 25670757PMC4457111

[7] ZhangJ, BaranJ, CrosA, GubermanJM, HaiderS, HsuJ, et al. International Cancer Genome Consortium Data Portal—a one-stop shop for cancer genomics data. Database. 2011;2011: bar026. doi: 10.1093/database/bar026 21930502PMC3263593

[8] HaendelMA, McMurryJA, RelevoR, MungallCJ, RobinsonPN, ChuteCG. A Census of Disease Ontologies. Annu Rev Biomed Data Sci. 2018;1: 305–331.

[9] WilkinsonMD, DumontierM, AalbersbergIJJ, AppletonG, AxtonM, BaakA, et al. The FAIR Guiding Principles for scientific data management and stewardship. Sci Data. 2016;3: 160018. doi: 10.1038/sdata.2016.18 26978244PMC4792175

[10] WilsonSL, WayGP, BittremieuxW, ArmacheJ-P, HaendelMA, HoffmanMM. Sharing biological data: why, when, and how. FEBS Lett. 2021;595: 847–863. doi: 10.1002/1873-3468.14067 33843054PMC10390076

[11] HaendelM, SuA, McMurryJ, ChuteCG, MungallC, GoodB, et al. Metrics to assess value of biomedical digital repositories: response to RFI NOT-OD-16-133. Geneva: Zenodo. 2016.

[12] Rubinstein YR, Robinson PN, Gahl WA, Avillach P, Baynam G, Cederroth H, et al. The case for open science: rare diseases. Jamia Open. [cited 16 Sep 2020]. doi: 10.1093/jamiaopen/ooaa030PMC766096433426479

The article "Phenopacket-tools: Building and validating GA4GH Phenopackets" was published in 2023. Journal: PLoS One.

[13] HuangB, TangY. Research on optimization of real-time efficient storage algorithm in data information serialization. PLoS One. 2021;16: e0260697. doi: 10.1371/journal.pone.0260697 34914712PMC8675695

[14] WhetzelPL, NoyNF, ShahNH, AlexanderPR, NyulasC, TudoracheT, et al. BioPortal: enhanced functionality via new Web services from the National Center for Biomedical Ontology to access and use ontologies in software applications. Nucleic Acids Res. 2011;39: W541–5. doi: 10.1093/nar/gkr469 21672956PMC3125807

[15] NadendlaS, JacksonR, MunroJ, QuagliaF, MészárosB, OlleyD, et al. ECO: the Evidence and Conclusion Ontology, an update for 2022. Nucleic Acids Res. 2022;50: D1515–D1521. doi: 10.1093/nar/gkab1025 34986598PMC8728134

[16] SioutosN, de CoronadoS, HaberMW, HartelFW, ShaiuW-L, WrightLW. NCI Thesaurus: a semantic model integrating cancer-related clinical and molecular information. J Biomed Inform. 2007;40: 30–43. doi: 10.1016/j.jbi.2006.02.013 16697710

[17] RobinsonPN, KöhlerS, BauerS, SeelowD, HornD, MundlosS. The Human Phenotype Ontology: a tool for annotating and analyzing human hereditary disease. Am J Hum Genet. 2008;83: 610–615. doi: 10.1016/j.ajhg.2008.09.017 18950739PMC2668030

[18] KöhlerS, GarganoM, MatentzogluN, CarmodyLC, Lewis-SmithD, VasilevskyNA, et al. The Human Phenotype Ontology in 2021. Nucleic Acids Res. 2021;49: D1207–D1217. doi: 10.1093/nar/gkaa1043 33264411PMC7778952

[19] 100,000 Genomes Project Pilot Investigators, SmedleyD, SmithKR, MartinA, ThomasEA, McDonaghEM, et al. 100,000 Genomes Pilot on Rare-Disease Diagnosis in Health Care—Preliminary Report. N Engl J Med. 2021;385: 1868–1880. doi: 10.1056/NEJMoa2035790 34758253PMC7613219

[20] DrenkhahnC, IngenerfJ. The LOINC Content Model and Its Limitations of Usage in the Laboratory Domain. Stud Health Technol Inform. 2020;270: 437–442. doi: 10.3233/SHTI200198 32570422

[21] MungallCJ, TorniaiC, GkoutosGV, LewisSE, HaendelMA. Uberon, an integrative multi-species anatomy ontology. Genome Biol. 2012;13: R5. doi: 10.1186/gb-2012-13-1-r5 22293552PMC3334586

[22] HuangQ, Carrio-CordoP, GaoB, PalootsR, BaudisM. The Progenetix oncogenomic resource in 2021. Database. 2021;2021. doi: 10.1093/database/baab043 34272855PMC8285936

[23] LadewigMS, JacobsenJOB, WagnerAH, DanisD, El KassabyB, GarganoM, et al. GA4GH phenopackets: A practical introduction. Advanced Genetics. 2022; 2200016. doi: 10.1002/ggn2.202200016 36910590PMC10000265

[24] ShefchekKA, HarrisNL, GarganoM, MatentzogluN, UnniD, BrushM, et al. The Monarch Initiative in 2019: an integrative data and analytic platform connecting phenotypes to genotypes across species. Nucleic Acids Res. 2020;48: D704–D715. doi: 10.1093/nar/gkz997 31701156PMC7056945

The article "Phenopacket-tools: Building and validating GA4GH Phenopackets" was published in 2023. Journal: PLoS One.

[25] CôtéR, ReisingerF, MartensL, BarsnesH, VizcainoJA, HermjakobH. The Ontology Lookup Service: bigger and better. Nucleic Acids Res. 2010;38: W155–60. doi: 10.1093/nar/gkq331 20460452PMC2896109

[26] OngE, XiangZ, ZhaoB, LiuY, LinY, ZhengJ, et al. Ontobee: A linked ontology data server to support ontology term dereferencing, linkage, query and integration. Nucleic Acids Res. 2017;45: D347–D352. doi: 10.1093/nar/gkw918 27733503PMC5210626

[27] NelsonSJ, ZengK, KilbourneJ, PowellT, MooreR. Normalized names for clinical drugs: RxNorm at 6 years. J Am Med Inform Assoc. 2011;18: 441–448. doi: 10.1136/amiajnl-2011-000116 21515544PMC3128404

[28] WishartDS, FeunangYD, GuoAC, LoEJ, MarcuA, GrantJR, et al. DrugBank 5.0: a major update to the DrugBank database for 2018. Nucleic Acids Res. 2018;46: D1074–D1082. doi: 10.1093/nar/gkx1037 29126136PMC5753335

[29] AvramS, BologaCG, HolmesJ, BocciG, WilsonTB, NguyenD-T, et al. DrugCentral 2021 supports drug discovery and repositioning. Nucleic Acids Res. 2021;49: D1160–D1169. doi: 10.1093/nar/gkaa997 33151287PMC7779058

[30] UrsuO, HolmesJ, BologaCG, YangJJ, MathiasSL, StathiasV, et al. DrugCentral 2018: an update. Nucleic Acids Res. 2019;47: D963–D970. doi: 10.1093/nar/gky963 30371892PMC6323925

[31] HastingsJ, OwenG, DekkerA, EnnisM, KaleN, MuthukrishnanV, et al. ChEBI in 2016: Improved services and an expanding collection of metabolites. Nucleic Acids Res. 2016;44: D1214–9. doi: 10.1093/nar/gkv1031 26467479PMC4702775

[32] GaultonA, HerseyA, NowotkaM, BentoAP, ChambersJ, MendezD, et al. The ChEMBL database in 2017. Nucleic Acids Res. 2017;45: D945–D954. doi: 10.1093/nar/gkw1074 27899562PMC5210557

[33] HeY, SarntivijaiS, LinY, XiangZ, GuoA, ZhangS, et al. OAE: The Ontology of Adverse Events. J Biomed Semantics. 2014;5: 29. doi: 10.1186/2041-1480-5-29 25093068PMC4120740

[34] Preston-Werner T. [No title]. [cited 30 Sep 2022]. Available: https://semver.org/

[35] ISO 4454:2022. In: ISO [Internet]. 2022 [cited 13 Oct 2022]. Available: https://www.iso.org/standard/79991.html

[36] RobinsonPN, RavanmehrV, JacobsenJOB, DanisD, ZhangXA, CarmodyLC, et al. Interpretable Clinical Genomics with a Likelihood Ratio Paradigm. Am J Hum Genet. 2020;107: 403–417. doi: 10.1016/j.ajhg.2020.06.021 32755546PMC7477017

[37] SmedleyD, JacobsenJOB, JägerM, KöhlerS, HoltgreweM, SchubachM, et al. Next-generation diagnostics and disease-gene discovery with the Exomiser. Nat Protoc. 2015;10: 2004–2015. doi: 10.1038/nprot.2015.124 26562621PMC5467691

[38] VorisekCN, LehneM, KlopfensteinSAI, MayerPJ, BartschkeA, HaeseT, et al. Fast Healthcare Interoperability Resources (FHIR) for Interoperability in Health Research: Systematic Review. JMIR Med Inform. 2022;10: e35724. doi: 10.2196/35724 35852842PMC9346559

The article "Phenopacket-tools: Building and validating GA4GH Phenopackets" was published in 2023. Journal: PLoS One.

[39] GA4GH Phenopacket Schema FHIR core-ig. Github; Available: https://github.com/phenopackets/core-ig

[40] BönischC, KesztyüsD, KesztyüsT. Harvesting metadata in clinical care: a crosswalk between FHIR, OMOP, CDISC and openEHR metadata. Sci Data. 2022;9: 659. doi: 10.1038/s41597-022-01792-7 36307424PMC9616884

[41] OverhageJM, RyanPB, ReichCG, HartzemaAG, StangPE. Validation of a common data model for active safety surveillance research. J Am Med Inform Assoc. 2012;19: 54–60. doi: 10.1136/amiajnl-2011-000376 22037893PMC3240764

[42] Núria Queralt-Rosinach, Pablo Alarcón, Tiffany Callahan, GiovanniDelussu, Charlotte Fraboulet, Romain Goussault, et al. Mapping OHDSI OMOP Common Data Model and GA4GH Phenopackets for COVID-19 disease epidemics and analytics. [cited 5 Apr 2023]. Available: https://biohackrxiv.org/ep3xh/

[43] SmedleyD, SchubachM, JacobsenJOB, KöhlerS, ZemojtelT, SpielmannM, et al. A Whole-Genome Analysis Framework for Effective Identification of Pathogenic Regulatory Variants in Mendelian Disease. Am J Hum Genet. 2016;99: 595–606. doi: 10.1016/j.ajhg.2016.07.005 27569544PMC5011059

